# Exogenous IL-4-Expressing Bone Marrow Mesenchymal Stem Cells for the Treatment of Autoimmune Sensorineural Hearing Loss in a Guinea Pig Model

**DOI:** 10.1155/2014/856019

**Published:** 2014-04-22

**Authors:** Chang-qiang Tan, Xia Gao, Lang Guo, He Huang

**Affiliations:** ^1^State Key Laboratory of Materials-Oriented Chemical Engineering, College of Biotechnology and Pharmaceutical Engineering, Nanjing University of Technology, No. 5 Xinmofan Road, Nanjing, Jiangsu 210009, China; ^2^Department of Otolaryngology-Head and Neck Surgery, Affiliated Nanjing Drum Tower Hospital of Nanjing University Medical School, Nanjing, Jiangsu 210008, China; ^3^Department of Otolaryngology, Nanjing Stomatological Hospital, Nanjing, Jiangsu 210008, China

## Abstract

Bone marrow mesenchymal stem cells (BMSCs) expressing recombinant IL-4 have the potential to remediate inflammatory diseases. We thus investigated whether BMSCs expressing exogenous IL-4 could alleviate autoimmune sensorineural hearing loss. BMSCs isolated from guinea pigs were transfected with recombinant lentivirus expressing IL-4. A total of 33 animals were divided into three groups. Group A received scala tympani injection of IL-4-expressing BMSCs, and Group B received control vector-expressing BMSCs, and Group C received phosphate-buffered saline. The distribution of implanted BMSCs in the inner ears was assessed by immunohistochemistry and fluorescence microscopy. Auditory brain-stem response (ABR) was monitored to evaluate the auditory changes. Following BMSCs transplantation, the threshold levels of ABR wave III decreased in Groups A and B and significant differences were observed between these two groups (P < 0.05). Transplanted BMSCs distributed in the scala tympani and scala vestibuli. In some ears with hearing loss, there was a decrease in the number of spiral ganglion cells and varying degrees of endolymphatic hydrops or floccule. Following transplantation, the lentivirus-infected BMSCs migrated to the inner ear and produced IL-4. Our results demonstrate that, upon transplantation, BMSCs and BMSCs expressing recombinant IL-4 have the ability to remediate the inflammatory injury in autoimmune inner ear diseases.

## 1. Introduction

Immune-mediated inner ear disease (IMIED), including local inflammatory diseases of the inner ear and autoimmune inner ear disease (AIED), often leads to inner ear tissue damage and physiological dysfunction. Such damage includes loss of sensorineural hearing and balance. The administration of immunosuppressive agents, such as adrenal corticosteroids and cytotoxic immunosuppressive agents, has been found to be effective in treating immune-inflammatory diseases; however, such treatments have been shown to have side effects, and, furthermore, the rate of relapse after drug withdrawal of such therapies is reported to be high [1]. Cavities in the inner ear facilitate local gene therapy as an alternative therapy that offers long-term benefits following administration of a single dose.

Bone marrow mesenchymal stem cells (BMSCs) are considered favorable vehicles for gene therapy owing to their multidifferentiation potential and their ability to migrate into sites of acute injury [2–7]. In vitro experiments have demonstrated long-term expression of exogenous genes delivered into BMSCs, thus making it possible to use genetically modified BMSCs for the treatment of diseases [8]. Compared with directly injected recombinant lentiviruses, transplanted BMSCs expressing desired exogenous genes from tailor-made lentiviruses allow for better control of the amount of genes introduced. When BMSCs transfected with recombinant lentiviruses are transplanted into the inner ear, the delivered therapeutic genes become concentrated at the lesions. In such cases, the amount of lentiviral vectors needed for the treatment is significantly lower, thus lowering the risk of adverse events. Numerous reports have demonstrated the therapeutic value of BMSCs [2, 7–11]. Furthermore, BMSCs play immunoregulatory roles and are involved in the genesis and progression of autoimmune diseases [12].

Interleukin-4 (IL-4), a cytokine secreted by T helper cell type 2 (Th_2_), stimulates the proliferation of B cells and T cells and promotes the differentiation of CD4^+^ T cells into Th_2_. IL-4 also plays key roles in the regulation of humoral and adaptive immunities. Similar to IL-10 and Fas L, IL-4 has anti-inflammatory effects; and IL-4, IL-10, IL-13, and other cytokines are secreted in large amounts to antagonize the inflammatory response when Th_2_ dominates in inflamed tissues. Genes encoding immunomodulatory molecules (such as IL-4, IL-10, soluble tumor necrosis factor receptor, chemokine antagonists, superoxide dismutase, and eliminating enzymes of reactive oxygen species) have been transduced into the joint cavity in order to antagonize the inflammation in rheumatoid arthritis and to induce a Th1 to Th2 immune shift. IL-4 has previously been administered via direct intramuscular or intra-articular injection of IL-4 plasmids or via infection with IL-4-recombinant adeno-associated viruses [13]. A separate study found that a combination of IL-4 and FasL had beneficial anti-inflammatory effects [14]. IL-4 was thus selected as the therapeutic gene for treating AIED in this study and we demonstrate here that BMSC-mediated delivery of IL-4 into the inner ear restores lost auditory function in guinea pig models of AIED.

Animal models of autoimmune sensorineural hearing loss (ASNHL) were generated by immunization of guinea pigs with PIEAg (58 kDa). BMSCs infected with recombinant lentivirus harboring the IL-4 gene, no-load BMSCs, and phosphate-buffered saline (PBS) were injected into the scala tympani of the inner ears of experimental animals. The distribution of transplanted cells, their immunomodulatory effects, and recovery from AIED are described.

## 2. Materials and Methods

### 2.1. Experimental Animals

Forty-four red-eyed white guinea pigs of either sex, aged 6–8 weeks and weighing 250–300 g, were used in this study and provided by the Experimental Animal Center of Nanjing Medical University. This study was carried out under strict adherence to the regulations on the management of laboratory animals, established by the State Scientific and Technological Commission of the People's Republic of China and the experimental protocol used was approved by the Committee on the Ethics of Animal Experiments, Nanjing Medical University (Permit Number: 2090560). All surgeries were performed under pentobarbital sodium or ether anesthesia and all efforts were made to minimize animal suffering. Prior to being subjected to experimental procedures, animals were shown to have normal auricle reflexes and were devoid of middle ear diseases as confirmed by otoscopy.

### 2.2. Preparation of Purified Inner Ear Antigen (PIEAg)

After ether anesthesia, guinea pigs were sacrificed by cervical dislocation and auditory vesicles were removed. The membranous labyrinth, including basement membrane, spiral ligament, semicircular tube, utricle, and saccule without otolith, was removed under a dissecting microscope and placed in 0.1 mol L^−1^ PBS (pH 7.4). After grinding, freezing, thawing, ultrasonication, homogenization, and centrifugation (×900 g), the supernatant was separated and inner ear tissue antigen (IETAg) was prepared. The protein content was indirectly estimated by using a UV-Vis spectrophotometer, and the protein solution was subpackaged. Nondenaturing gel electrophoresis was used to separate proteins contained in IETAg. The 58-kDa band was excised from the gel, ground up, and homogenized for preparation of PIEAg [15].

### 2.3. Construction of an ASNHL Animal Model

PIEAg gel homogenate (0.2 mL acquired from electrophoresis of 400 *μ*g IETAg) was emulsified with an equal volume of complete Freund's adjuvant (Sigma, USA) and subcutaneously injected into the right rear foot pads and multipoints in backs of animals. Subsequently, half the first dose of PIEAg with an equal volume of incomplete Freund's adjuvant (Sigma, USA) was injected two weeks and four weeks after the initial immunization to strengthen the immune response.

Two weeks after the last immunization, if the thresholds of the auditory brain-stem response (ABR) wave III were higher than the sum of the mean value and twice the standard deviation in preimmunized animals, and if PIEAg-specific antibodies were detected, the ASNHL animal model was considered to have been successfully generated. PIEAg-specific antibodies were quantitated by ELISA. Samples were considered positive for PIEAg-specific antibodies if the absorbance at 490 nm was higher than the mean absorbance value plus 2 times the standard deviation ($\overset{-}{A}\pm \text{SD}$) in preimmunized animals. A total of 33 model animals were generated.

### 2.4. Isolation, Culture, and Labeling of BMSCs

#### 2.4.1. Separation of Femur

Red-eyed white guinea pigs aged 3-4 weeks and weighing 250–300 g were anesthetized with ether, soaked in 75% alcohol for 20 min, and sacrificed by cervical dislocation. The skin and muscle of the thigh were cut in order to expose the femur. Femurs on both sides of each animal were separated and placed for 5 min in a petri dish containing sterilized PBS.

#### 2.4.2. Isolation and Culture of BMSCs

5 mL Dulbecco's Modified Eagle's Medium (DMEM, low glucose) containing 10% fetal bovine serum was added to a petri dish. The two ends of the femur were removed, after which the bone marrow was flushed out using a 5 mL syringe and serum-free medium until the color of femur turned white in color. The marrow from both femur bones of the same guinea pig was pooled, mixed by repeated syringing, transferred to a 10 mL centrifuge tube, and centrifuged at ×900 g for 10 min. The supernatant and fat layer were discarded. L-DMEM containing 10% fetal bovine serum, 1% penicillin, and 1% streptomycin was added to the cell pellet. After counting, the cells were seeded in a 25 cm^2^ culture flask at a concentration of 1 × 10^6^ cells/mL with 15 mL culture medium.

#### 2.4.3. Culture and Passage

Cells were cultured in a humidified incubator at 5% CO_2_ and 37°C for 48 h, after which spent medium was replaced with fresh culture medium. Culture medium was subsequently changed every 3 or 4 days. At 80%–90% confluence, cells were digested with 0.25% trypsin and passaged at a 1 : 2 ratio.

#### 2.4.4. Harvesting BMSCs

Guinea pig BMSCs were separated using a previously described adherence method with modifications [16, 17] and were cultured in DMEM. The main difference from the traditional method is that we shortened the interval of changing cell medium in the early primary culture, 3 h for the first time and 8 h for the rest of times. This can greatly remove the contaminating cells-hematopoietic stem cells (HSCs). The digestive time by trypsin was shortened from 5~6 min to 2 min in order to avoid reducing the activity of MSCs. After 3 passages, BMSCs were obtained at high purity ready for lentiviral infection (shown in Figure 1).

### 2.5. Packaging of Lentiviral Vector and Validation of Recombinant Lentivirus

#### 2.5.1. Packaging and Labeling of Lentiviral Vector

The envelope plasmid (pVSG), the packaging plasmid (pHELPER), and vector plasmid (pNL-IRES2.EGFP) were mixed at a ratio of 1 : 1 : 1 (total: 8 mg). High-glucose DMEM was added at a final volume of 0.5 mL, and the solution was mixed briefly. Lipofectamine 2000 (20 *μ*L) was diluted into 0.5 mL with the high-glucose DMEM and mixed with the solution containing plasmids. After the mixture was incubated for 5 min at room temperature, it was added to 293T cells in a 60 mm petri dish. The cells were cultured at 37°C under 5% CO_2_ in a humidified incubator for 6 h, after which, the culture medium was removed, complete growth medium was added, and the culture was further incubated. Cells were examined under a fluorescence microscope at 24 h after transfection. At 48 h and 72 h after transfection, the supernatant containing virus was harvested and centrifuged at ×2800 g for 20 min. The supernatant was collected and stored at −70°C (provided by Shanghai Dior Biological Research Institute).

#### 2.5.2. Validation of Lentivirus pll3.7-IL-4

2 mL pll3.7-IL-4 lentivirus solution was added to 293T cells at 80% confluence. Cells were harvested when most cells had a rounded appearance and still were adherent. Lentivirus particles were releaved from cells by three cycles of freezing and thawing, after which lentiviral DNA was extracted for polymerase chain reaction (PCR) validation (Figure 2). PCR result confirmed the presence of the rat IL-4 CDS-X2746G in lentiviral DNA.

### 2.6. Infection of BMSCs with Lentivirus

BMSCs (passage 3) grown to 80% confluence in a 25-cm^2^ cell culture flask were infected with 15 *μ*L recombinant lentivirus (1 × 10^8^ particles/mL). Polybrene reagent was then added at a final concentration of 8 mg/L. After 8 h, the medium was replaced with complete medium. At 24 h after infection, the cells were examined under a fluorescence microscope. The infection procedure was repeated to reinfect the BMSCs. 48 h after the first infection, the expression of green fluorescent protein was assessed using fluorescence microscopy. Bright yellow-green fluorescence indicated successful infection (Figure 3). Infected BSMCs were passaged at 90% confluence. Lentiviral transduction was further analyzed by PCR by using cDNA prepared from infected BMSCs (Figure 4). The primers used for PCR amplification of IL-4 were 5′-GCTAT-TGATGGGTCTCACCC-3′ (F) and 5′-CAGGACGTCAAGGTA-CAGGA-3′ (R) and yielded a PCR product of 412 bp. The annealing temperature used for PCR was 60°C. A similar protocol using no-load lentivirus (lentivirus not containing IL-4 CDS) was followed for preparing no-load BMSCs. Successfully infected BMSCs were used for transplantation.

### 2.7. Grouping and Implantation of BMSCs

#### 2.7.1. Grouping

The 33 animals, modeling ASNHL, were divided into 3 groups with a paired design. Suspension of BMSCs infected with recombinant lentivirus harboring IL-4 was injected into the inner ears of guinea pigs in Group A. Suspension of BMSCs infected with no-load lentivirus was injected into the inner ears of guinea pigs belonging to group B. PBS was injected into the inner ears of Guinea pigs in Group C. The volume injected was 20 *μ*L in each group. The cell density in BMSCs suspensions was approximately 1.5–2.0 × 10^10^ L^−1^.

#### 2.7.2. Implantation of BMSCs into the Inner Ear

Successfully infected BMSCs (P3) were digested with trypsin, centrifuged at 1000 r× min^−1^ for 10 min, and resuspended in DMEM. After cell counting, cell concentration was adjusted to 1.0–2.0 × 10^10^ L^−1^. Two weeks after the last immunization, guinea pigs were anesthetized by intraperitoneal injection of 1% pentobarbital sodium (30 mg/kg). An arc incision of 2-3 cm in length was made behind the pinna. Subcutaneous muscle and fascia were separated to expose the bulla. Using a microelectric drill, the bulla was opened to expose basal turn of cochlea. A hole was drilled on the bone wall of the scala tympani to accommodate a needle, avoiding penetration of the inner periosteum. A scalp needle was inserted into scala tympani by using a microthruster at a depth less than 1 mm. A small volume of perilymph was extracted (about 10 *μ*L). Following this, BMSC suspensions or PBS was slowly injected into the scala tympani by using a microinjection machine. The hole in the cochleostomy was closed with bone wax, and the middle ear cavity was flushed three times with an antibiotic solution. The hole in the bulla was then closed with bone wax. The incision was sutured by layer. All manipulations were performed under sterile conditions.

### 2.8. Observational Indexes

#### 2.8.1. Assay of Specific Antibodies in Serum

Blood samples were collected by cardiac puncture method at three time points—before immunization, 2 weeks after the last immunization, and 1 week after scala tympani implantation. Serum was separated from the whole blood. The serum levels of specific antibodies against PIEAg were determined by ELISA. Gel homogenate of PCIEAg (100 *μ*g/mL) was used to coat ELISA plates (100 *μ*L/well), and they were incubated at 4°C overnight. The plate was washed 3 times with PBST for 5 min each. Serum from animals diluted with PBS at a ratio of 1 : 10 (100 *μ*L/well) was added, and the plate was incubated at 37°C for 2 h. The plates were washed 3 times with PBST. Horseradish peroxidase-labeled goat anti-guinea pig IgG polyclonal antibody (Sigma, USA) diluted at a ratio of 1 : 2000 (100 *μ*L well) was added, and the plate was incubated at 37°C for 1 h. After washing with PBST, 3,3,5,5-tetramethyl benzidine (TMB) was added and plate was incubated at 37°C for 10 min. The reaction was terminated with 2 mol/L H_2_SO_4_. The absorbance at 490 nm was measured by enzyme-linked immunometric meter.

#### 2.8.2. Auditory Brain-Stem Response (ABR) Test

Auditory function was tested by Tucker Davis Technology (TDT) BioSig System III (TDT system 3) (TDT Company, American) before immunization, 2 weeks after the last immunization, and 1 week after BMSC transplantation. A needle electrode was inserted into the head of the animals as the test electrode at the junction of coronal and sagittal sutures. A reference electrode was placed near the mastoidale on the rear side of the pinna. The grounding electrode was placed on the tip of the nose. The acoustic stimulus signal was a Click. The repetition frequency was 11 times per second. Recording period was 10 ms. The threshold of ABR wave III was determined (dB, SPL).

#### 2.8.3. Pathomorphological Observation of Inner Ear

Guinea pigs were sacrificed by cervical dislocation after ether anesthesia (2 animals), 2 weeks after the last immunization (2 animals), and 1 week after BMSC transplantation (2 animals). The temporal bone was removed immediately. The bulla (otic vesicle) was opened and placed in 4% paraformaldehyde for 12 h and later in 10% ethylenediaminetetraacetic acid (EDTA) for 5–7 days for decalcification. After trimming, it was flushed with running water for 1-2 h, dehydrated, made transparent, wax dipped, and embedded. Slices of 5 *μ*m thickness were cut through the central axis of cochlea. The sections were rinsed with distilled water and dried upright in order to facilitate adhesion between the section and the charged glass surface. Standard hematoxylin and eosin (H&E) staining was performed on mounted sections, after which sections were examined under a light microscope and photographed.

#### 2.8.4. Immunohistochemistry

*Embedding Inner Ear in Paraffin and Sectioning*. One week after BMSC transplantation, the rest of the guinea pigs in each group were sacrificed by cervical dislocation following anesthesia. The temporal bone was immediately removed, and the bulla was opened and placed in 4% paraformaldehyde. The round window was opened with a needle. A small hole was drilled in the apex of the cochlea, which was then infused rapidly with 4% paraformaldehyde and fixed for 12 h. Following decalcification with EDTA for 1 week, trimming, and flushing with running water for 1 h, the tissue was dehydrated, made transparent, wax dipped, and embedded.

*Fluorescence Autography*. Cochlear central axis slices (5 *μ*m thickness) were prepared from 4 guinea pigs belonging to each group. The sections were rinsed with distilled water, dried upright, dewaxed with water, examined using a fluorescence microscope, and photographed.

*Immunohistochemistry*. Paraffin-embedded sections of cochlea were prepared from 3 animals (6 ears) from each group as described before. Antigen retrieval was performed with 0.2% trypsin. Sections were blocked with normal goat serum for 10 min. First, antibody (rabbit anti-mouse IL-4 monoclonal antibody) diluted in PBS was added, and sections were incubated at 4°C overnight. Following this, the sections were rinsed 3 times with PBS for 5 min each. HRP-conjugated goat anti-rabbit IgG monoclonal antibody was added, and the sections were incubated at 37°C for 30 min. After rinsing 3 times with PBS, the sections were stained with DAB (3,3′-diaminobenzidine) and mounted with resin. The slides were examined under a light microscope and photographed.

## 3. Results

### 3.1. Specific Immune Response Test

As shown in Table 1, the levels of specific antibodies raised against PIEAg increased significantly after immunization in the experimental group and control groups (paired *t*-test, mean of left and right ear, *P* < 0.05). No significant differences were observed among different groups before and after immunization (paired* t*-test, mean of left and right ear, *P* > 0.05) and no significant differences were observed between the antibody levels detected after immunization and those detected after the transplantation of cells (*P* < 0.05).

### 3.2. Auditory Functions

The ABR wave III threshold was used as the indicator to assess hearing, and the results of these assessments are shown in Table 2. Compared with those before immunization, the average thresholds of ABR wave III in each group increased significantly after immunization (*t*-test, *P* < 0.05). When compared to those after immunization with PIEAg, the average thresholds of ABR wave III in Groups A and B decreased significantly after local injection of BMSCs into the inner ear (*t*-test, *P* < 0.05)—more significantly in Group A. The average threshold of ABR wave III in Group C showed no significant change after local injection of PBS into the inner ear. There were no significant differences in the average threshold of ABR wave III between the left ears and right ears in each group over the same period (*t*-test, *P* > 0.05). After local injection into the inner ear, if the threshold of ABR wave III in an animal was lower than the average threshold value detected after immunization minus two times standard deviations, its auditory functions were considered to have improved. Auditory functions improved in 7 cases (12 ears) of Group A and 5 cases (9 ears) of Group B—the effective rates were 54.55% (12 ears/22 ears) and 40.91% (9 ears/22 ears), respectively. However, no improvement was observed in the auditory functions of the animals in Group C.

### 3.3. Examination of the Inner Ear by Light Microscopy

As shown in Figures 5(a)–5(d), inflammatory reactions in the inner ears of animals were evident in each group after immunization. This included infiltration of inflammatory cells (mainly mononuclear cells) in Rosenthal's tube and the spiral ganglion, degeneration (mainly displayed as cell swelling) and decrease of spiral ganglion cells, visible flocs in cochlear duct, scala tympani, or scala vestibule, blood in the scala tympani, and “floating cells” in the cochlear duct. No obvious abnormalities were observed in the morphologies of the organ of Corti and hair cells. After the transplantation of BMSCs, the inflammatory reactions in Groups A and B were significantly milder than those in the control group (Group C), particularly so in the case of ears with improved auditory function—mononuclear cell infiltration was observed only around the modiolar blood vessels; the morphology and numbers of spiral ganglion cells were normal; and no evident abnormalities in the organ of Corti and stria vascularis were observed. Flocs were observed in some scala tympani, but “floating cells” were not found.

### 3.4. Fluorescence Autography

In Groups A (Figure 6(a)) and B (Figure 6(b)), intense fluorescence from clumps of cells was observed in the scala tympani and scala vestibule after BMSC transplantation. Fluorescence was also observed in the stria vascularis, the lips of the osseous spiral lamina, and the organ of Corti, as well as under the vestibular membrane. No obvious fluorescence was detected in samples from Group C (Figure 6(c)).

### 3.5. Immunohistochemistry

After IHC, cell clumps in the scala tympani and the lips of the osseous spiral lamina of animals in Group A showed obvious brown color (Figures 7(a) and 7(b)), indicating that enzyme reactions were positive. The organ of Corti and spiral ganglion showed weak staining. In group B (Figure 7(c)), no evidence of positive enzyme reactions in cell clumps in the scala tympani or other parts of the inner ear was found. In Group C (Figure 7(d)), no evidence of positive enzyme reactions was found in the inner ear.

## 4. Discussion

ASNHL was first reported by McCabe in 1979 [18], and, since then, a class of diseases caused by immune-mediated inner ear damage have been reported. These conditions have been collectively called IMIED and include AIED, immune-mediated bilateral Meniere's disease, and inner ear diseases caused by systemic autoimmune diseases. The etiology and pathogenesis of immune injury-related inner ear diseases remain unclear, and corticosteroids and immunosuppressive agents have therefore been used in the treatment of IMIED. Although this treatment strategy is successful during the early period, numerous side effects and rapid relapse following drug withdrawal are commonly reported. Cavities in the inner ear facilitate local injection of drugs and, compared with systemic administration, local treatment offers four major advantages [19–22]: (1) improved targeting; (2) delivery directly into the inner ear, avoiding blood labyrinth barrier; (3) higher drug concentration in endolymph and perilymph; and (4) reduced systemic drug toxicity and minimizing side effects.

The blood labyrinth barrier serves to maintain a stable liquid labyrinth when blood components change in response to the changes of the systemic conditions. Drugs administered systemically can pass through this barrier into the local capillaries, and then through endolymphatic or perilymphatic the cavity go into the important structures of the inner ear such as organ of Corti. This barrier is able to limit many drugs passing into the inner ear. However, administration through the inner ear (including the inner ear window, the round window membrane permeation, and the lymph sac injections) can avoid this barrier, so that drugs concentrate locally to achieve effective treatment concentration. In clinical practice, taking into account the risk of damage to the inner ear via the inner ear window, the round window membrane permeation or the sac injections are preferred.

In our previous studies, we demonstrated that local injection of drugs into the inner ear does not lead to any significant physiological dysfunction of the inner ear. We found that direct administration of adenovirus or lentivirus carrying therapeutic genes into the inner ear had a therapeutic effect on autoimmune sensorineural hearing loss [23]. Controlling the amount of virus delivered to the inner ear, however, has proven to be a difficult task. Additionally, the safety of administering adenovirus and lentivirus directly to the inner ear is still contested. Cells, including BMSCs, have been used effectively as alternate vehicles for introducing therapeutic genes to the inner ear [24].

BMSCs exhibit multidirectional differentiation potential, immunosuppressive function, and low immunogenicity. Furthermore, BMSCs have been shown to be useful for the treatment of inner ear inflammatory damage. Sharif et al. [25] showed that BMSCs carrying the enhanced green fluorescent protein (EGFP) gene transplanted into the inner ear of healthy C57BL/6 mice migrated to the cochlea. Despite the distribution of transplanted cells in the perilymphatic space, fluorescence was also detected in the spiral ligament and spiral limb, which was consistent with the fluorescence distribution observed in our study. Since some of the transplanted cells expressed connexin-26, these authors suggested that BMSCs might be used to transfer therapeutic molecules and repair cochlear cells, particularly near the spiral ligament and the spiral limb.

Many immune system-related diseases are characterized by hyperactivation of B lymphocytes and the production of large amounts of autoantibodies. Th2 cells secrete cytokines, including IL-4, IL-6, and IL-10. IL-4 stimulates the proliferation of T cells and B cells and studies [26] have shown that IL-4 stimulates human mononuclear cells to produce IL-1 receptor antagonist (IL-1Ra), which, in turn, inhibit the colony formation and migration of macrophages. IL-4 therefore plays a crucial role in controlling inflammation. In our study, we found that guinea pigs immunized with PIEAg and Freund's adjuvant were shown to suffer from sensorineural hearing loss. This was accompanied by an increase in serum levels of specific antibody against PIEAg, indicating the successful establishment of an animal model of ASNHL.

Recombinant lentiviral vectors harboring the IL-4 gene and a GFP reporter were constructed and used to infect BMSCs isolated from femoral shaft of guinea pigs. BMSCs infected with recombinant lentivirus produced IL-4 after transplantation into the inner ear of guinea pigs. Transplanted BMSCs were identified alive in the inner ear (primarily localized in scala tympani and scala vestibuli, with a few migrating to the organ of Corti, stria vascularis, and lip of the osseous spiral lamina), suggesting that, due to their low immunogenicity, BMSCs effectively avoided immune rejection. The results of immunohistochemistry experiments performed on samples from Groups B and C confirmed that the local IL-4 production in the inner ear induced by inflammation (background) was low. However, in Group A, cell clumps in the scala tympani, scala vestibule, and the lips of the osseous spiral lamina were strongly positive for IL-4, while the organ of Corti and spiral ganglion showed only weak staining. We thus conclude that elevated levels of IL-4 were produced by IL-4 gene-modified BMSCs after implantation into the inner ear. The results of immunohistochemistry and morphological analyses demonstrated that the inflammatory reactions in Groups A and B (particularly in the ears with improved auditory functions) were significantly milder than those in the control group (Group C). Auditory test results showed that the average thresholds of ABR wave III in Groups A and B dropped after transplantation of BMSCs, more significantly in Group A. Our findings confirmed that BMSCs may be used as a vehicle to deliver IL-4 to the sites of inner ear injury and that IL-4 delivered in this way facilitates recovery from autoimmune-mediated inner ear diseases by exerting its anti-inflammatory and immunomodulatory effects.

In this study, BMSCs expressing exogenous IL-4 were transplanted into the inner ear of guinea pigs by scala tympani injection. The results showed that transplanted BMSCs were broadly distributed in the inner ear. Based on the results, we hypothesize that BMSCs may be distributed in the cochlear duct through three distinct mechanisms: (1) transport through the small hole in the osseous spiral lamina to the perilymph of the scala tympani; (2) transport through the pores in which cochlear nerve fibers pass through to the perilymph of the scala tympani; (3) transport between the scala tympani and the scala vestibule through the helicotrema and the endolymph. Further studies are warranted to understand the distribution of BMSCs in the inner ear following scala tympani injection.

## Figures and Tables

**Figure 1:** BMSC morphology in culture. BMSCs (passage 3) observed under an inverted microscope (×100); uniform spindle-shaped BMSCs fused into a spiral shape.

**Figure 2:** Validation of lentivirus pll3.7-IL-4. (a) Diagram of lentivirus pll3.7-IL-4. (b) Recombinant lentivirus pll3.7-IL-4 DNA digested with* Hind*III enzyme (left lane) compared with molecular marker bands (right lane). Gene name: rat IL-4 CDS-X2746G; clone ID#: D6466-2 RES:HindIII. Primers used for PCR amplification of IL-4 were 5′-GCTATTGATGGGTCTCACCC-3′ (F) and 5′-CAGGACGTCAAGGTACAGGA-3′ (R). The expected length of the PCR product was 412 bp and the annealing temperature used in PCR reactions was 60°C.

**Figure 3:** Fluorescence microscopy of BMSCs following infection with lentivirus. Fluorescence micrograph of Group A, Group B, and Group C BMSCs 48 h after infection with lentivirus (×200). Green fluorescence was observed in Group A (a) and Group B (b) but not in Group C (c).

**Figure 4:** RT-PCR analysis of lentiviral DNA. (a) PCR detection of lentiviral vector genes from BMSCs infected with lentivirus. DNA or cDNA served as templates for PCR and the expected length of the PCR product was 412 bp. Lane A: positive control; lane B: DNA from BMSCs infected by lentivirus vector; lane C: cDNA from BMSCs infected with lentivirus vector. (b) A lentivirus concentrate was used as a template for PCR detection of the lentiviral vector gene (lanes D1 and D2). M: DNA molecular markers.

**Figure 5:** Immunohistochemical assessment of inflammatory reactions in the inner ears of experimental animals. (a) Vertical slice of the cochlea from a guinea pig in Group C after immunization (40 × 10); RBCs and WBCs were detected in the scala tympani (indicated by the arrow). (b) Vertical slice of the cochlea from a guinea pig in Group B after transplantation of BMSCs into the inner ear (40 × 10); floccules were observed in the scala tympani (indicated by the arrow). (c) Vertical slice of the cochlea from a guinea pig in Group C after immunization (40 × 10); infiltration of inflammatory cells was observed in spiral ganglion (indicated by the arrow). (d) Vertical slice of the cochlea from a guinea pig in Group A after transplantation of BMSCs into the inner ear (40 × 10); the structure of the spiral ganglion was normal.

**Figure 6:** Fluorescence microscopic assessment of inner ear tissue following immunization of experimental animals. (a) One week after transplantation of BMSCs, cell clumps emitting intense fluorescence were observed in the scala tympani of a guinea pig in Group A (indicated by the arrow) (ST: scala tympani). (b) One week after transplantation of BMSCs, cell clumps emitting intense fluorescence were observed in the scala tympani of a guinea pig in Group B. Fluorescence could also be detected in stria vascularis and vestibular membrane (indicated by the arrows). (c) Absence of fluorescent cells in scala tympani of a guinea pig from Group C, 1 week after injection with PBS. ST: scala tympani.

**Figure 7:** (a, b) Vertical slices of cochlea in Group A (20 × 10); clumps of cells colored brown in scala tympani could be seen, indicating positive enzyme reactions. The lips of the osseous spiral lamina also showed positive staining (indicated by the arrow). (c) Vertical slice of cochlea from a guinea pig in Group B (10 × 10); clumps of cells were seen in scala tympani (indicated by the arrow). Neither the clumps of cells nor any other parts of the inner ear were stained brown. (d) Vertical slice of cochlea from a guinea pig in Group C; brown staining was not seen. Scattered blood cells in scala tympani were a result of the bleeding during the injection (indicated by the arrow).

**Table 1:** Serum levels of PCIEAg-specific antibody before and after immunization and after local injection into the inner ear (*A* value, $\overset{-}{\chi }\pm S$).

Groups	Before immunization	After immunization	After injection into the inner ear
Group A	0.4231 ± 0.0475	0.6683 ± 0.0371	0.6587 ± 0.0236
Group B	0.4345 ± 0.0453	0.6506 ± 0.0284	0.6468 ± 0.0352
Group C	0.4412 ± 0.0435	0.6649 ± 0.0403	0.6528 ± 0.0416

**Table 2:** The average thresholds of ABR wave III before and after immunization and after local injection into the inner ear (dB, SPL) ($\overset{-}{\chi }\pm 2S$).

Groups	Before immunization		After immunization		After injection into the inner ear	
	Left ear	Right ear	Left ear	Right ear	Left ear	Right ear
Group A	32.00 ± 5.70	34.00 ± 6.50	65.00 ± 5.40	71.00 ± 5.75	46 ± 7.00	45 ± 6.00
Group B	33.00 ± 6.80	32.00 ± 7.00	69.00 ± 7.30	70.00 ± 8.65	54 ± 6.53	54 ± 6.50
Group C	35.00 ± 6.70	34.00 ± 6.20	68.00 ± 7.50	71.00 ± 8.26	67 ± 8.50	69 ± 9.00
